The article "Blockchain-Based Encryption Method for Internal and External Health Privacy Data of University Physical Education Class" was published in 2022. Journal: J Environ Public Health.

# Blockchain-Based Encryption Method for Internal and External Health Privacy Data of University Physical Education Class

**DOI:** 10.1155/2022/7506894

**Published:** 2022-08-29

**Authors:** Zheng Zhou, Yang Liu

**Affiliations:** ^1^Hulunbuir University, Institute of Physical Education, Hulunbuir 021008, Inner Mongolia, China; ^2^Physical Education Institute of Shaanxi Normal University Shanxi, Xi'an 710119, China

## Abstract

In order to improve the security of the storage and scheduling of health privacy data inside and outside the university physical education class, a storage and scheduling method based on blockchain hybrid encryption is proposed. The distribution structure model of health privacy data blockchain inside and outside the university physical education class is established, arithmetic coding and quantitative feature analysis methods to schedule and adaptively control health privacy data blockchain inside and outside the university physical education class are adopted, public key coding configuration and vector quantization coding methods are combined to design encryption keys in the process of health privacy data transmission inside and outside the university physical education class, and blockchain hybrid encryption algorithm is adopted to design encryption keys for health privacy data inside and outside the university physical education class. The arithmetic coding is embedded in the encryption system, and the bit sequence output by the blockchain hybrid encryption is circularly shifted, so as to realize the encryption of health privacy data inside and outside the university physical education class and optimize the storage scheduling. The simulation results show that this method has good security encryption performance, strong antiattack ability, and balanced storage space allocation, which improves the security storage and transmission ability of health privacy data inside and outside the university physical education class.

## 1. Introduction

With the rapid increase in network communication data, people pay more attention to storage and scheduling of health privacy data inside and outside physical education classes, but in this process, network attack and virus intrusion will lead to leakage of health privacy data inside and outside physical education class, and the output security is not good. This article constructs a storage and scheduling model of health privacy data inside and outside the physical education class, through coding modulation and key control methods. To realize the storage and scheduling of health privacy data inside and outside the university physical education class, data encryption and arithmetic coding methods are combined and the security storage and information encryption model of health privacy data inside and outside the university physical education class is established [1]. Based on the design of dynamic encryption algorithm of health privacy data inside and outside the university physical education class, combined with dynamic data storage scheme, the security of health privacy data collection inside and outside the university physical education class is improved. The related research on storage and scheduling methods of health privacy data inside and outside the university physical education class has attracted great attention [2].

The article "Blockchain-Based Encryption Method for Internal and External Health Privacy Data of University Physical Education Class" was published in 2022. Journal: J Environ Public Health.

The storage and scheduling of health privacy data inside and outside the university physical education class is based on the coding and key control of communication encryption data. Nonlinear feature encryption method is adopted to control the storage and scheduling of health privacy data inside and outside the university physical education class. The traditional methods are mainly BPSK modulation method and chaotic mapping encryption method. Homomorphic mapping encryption method is adopted to control the storage and scheduling of health privacy data inside and outside the university physical education class. In reference [3], a revocable attribute-based encryption algorithm for Internet of Things based on blockchain is proposed, which uses blockchain model analysis and subspace noise reduction reorganization to realize multichannel secure encryption and transmission of health privacy data inside and outside the physical education class. However, this method has poor antiattack ability for multichannel encryption of health privacy data inside and outside the physical education class. In reference [4], a reversible steganography scheme of video encryption domain based on vector histogram migration is designed, and the encrypted transmission of video information is realized through histogram reconstruction, but this method has a large amount of computation and poor stability. To solve the above problems, this article proposes a storage and scheduling method of health privacy data inside and outside the university physical education class based on blockchain hybrid encryption. First, the distribution structure model of health privacy data blockchain inside and outside the university physical education class is established, and the blockchain scheduling and adaptive control of health privacy data inside and outside the university physical education class are carried out by arithmetic coding and quantitative feature analysis. The encryption key design in the process of health privacy data transmission inside and outside the university physical education class is combined with public key coding configuration and vector quantization coding method. Finally, the simulation test shows the superior performance of this method in improving the storage and scheduling ability of health privacy data inside and outside the university physical education class.

The article "Blockchain-Based Encryption Method for Internal and External Health Privacy Data of University Physical Education Class" was published in 2022. Journal: J Environ Public Health.

## 2. Multichannel Model and Data Characteristics Analysis of Health Privacy Data inside and outside Universities in Physical Education Class

### 2.1. Multichannel Model of Health Privacy Data inside and outside the University Physical Education Class

In recent years, the research on the current situation of college students' physical exercise has been fruitful, such as the current situation of physical exercise; the relationship between physical exercise and mental health; physical health, social health, and physique; and the research on college students' attitude, motivation, and habit of physical exercise.

In order to realize the storage and scheduling of health privacy data inside and outside the university physical education class based on blockchain hybrid encryption, first, a multichannel model of health privacy data inside and outside the university physical education class is constructed and the channel output carrier sequence of health privacy data inside and outside the university physical education class is analyzed by using channel equalization method. Channel equalization is an antifading measure taken to improve the transmission performance of communication systems in fading channels. It is mainly to eliminate or weaken the problem of intersymbol interference (ISI) caused by multipath delay in broadband communication. Combined with nonlinear dynamics and statistical physics theory [5], under the background of noise interference, filtering suppression method is adopted.

Digital filter can be divided into two parts: classical filter and modern filter. Classical filter assumes that the useful component and the desired component in the input signal *x*(*n*) are located in different frequency bands, so we can filter the noise through a linear system. If the spectrum of the noise and the signal are mixed, classical filter cannot meet the filtering requirements. There are usually high-pass filter, low-pass filter, band-pass filter, and band-stop filter. Modern filters estimate useful signals and noise signals from noisy signals. In this method, both signal and noise are regarded as random signals, and the signal estimation algorithm is derived by using its statistical characteristics, such as autocorrelation function, cross-correlation function, self-power spectrum, and cross power spectrum, which is then implemented by digital equipment. There are mainly Wiener filter, Kalman filter, and adaptive filter, along with other digital filters.

The article "Blockchain-Based Encryption Method for Internal and External Health Privacy Data of University Physical Education Class" was published in 2022. Journal: J Environ Public Health.

Classical filtering is an engineering concept based on Fourier analysis and transform. According to the theory of advanced mathematics, any signal that meets certain conditions can be regarded as the superposition of infinite sine waves. In other words, the engineering signal is a linear superposition of sine waves of different frequencies. Sine waves of different frequencies that make up the signal are called frequency components or harmonic components of the signal. In fact, any electronic system has its own bandwidth (the limit on the maximum frequency of the signal), and the frequency characteristic reflects the basic characteristic of the electronic system. The filter is an engineering application circuit designed according to the influence of circuit parameters on the circuit bandwidth. The modern filtering idea is quite different from the classical filtering idea. Modern filtering takes advantage of the randomness of the signal, regards the signal and its noise as random signals, and estimates the signal itself by using its statistical characteristics. Once the signal is estimated, the signal itself is much higher than the original signal-to-noise ratio. Typical digital filters include Kalman filter, Wenner filter, adaptive filter, wavelet transform, and other means. In essence, digital filtering is actually an algorithm that can be implemented on digital devices. These digital devices include not only computers, but also embedded devices such as DSP, FPGA, and arm. Digital filtering has the advantages of high precision, high reliability, programmable change of characteristics or multiplexing, easy integration, and so on. Digital filtering has been widely used in language signal processing, image signal processing, medical biological signal processing, and other application fields. Digital filtering includes low pass, high pass, band pass, band stop, and all pass. It can be time invariant or time-varying, causal or noncausal, linear or nonlinear. The most widely used is linear, time-invariant digital filter. The cepstrum eigenvalues of the health privacy data output inside and outside the university physical education class contain a subset of features, assuming that (*i*, *j*) is the correlation statistical eigenvalue of the health privacy data channel balance control inside and outside the university physical education class, which is the correlation degree between multiple orthogonal subchannels defining the orientation constraint eigenvalues of the main lobe of the array pattern. The process of array mode is shown in Figure 1.

The article "Blockchain-Based Encryption Method for Internal and External Health Privacy Data of University Physical Education Class" was published in 2022. Journal: J Environ Public Health.

The distribution set of coding links between the array suppression grating lobe and the signal bandwidth is obtained as Co(*r*). Under the condition of blockchain hybrid encryption, based on digital beam forming grating lobe, the spatial sampling frequency parameter *KC* ∈ {0,1,……, *n* − 1} after digital beam forming grating lobe is obtained, and the broadband true delay energy pattern is constructed in the achievable rate domain *S*_*i*_={(*j*, *i*, *k*)}. The broadband true delay energy construction process is shown in Figure 2.

The shift number of the signal received by the nth array element, with the minimum number of bits being ⌈log_2_(*n*)⌉ bits, establishes the distribution structure model of the health privacy data blockchain inside and outside the university physical education class, and the normal characteristic quantity of the broadband signal incident on the array element is obtained asCo(*r*) [6, 7] . Under optimal position and speed of channel transmission, by using symmetric coding and nonlinear encryption methods, the parameters of the side-grid suppression structure model of the kth cycle are obtained as *e*_*S*_*i*__^*t*^=*e*_*ik*_^*t*^. The three-dimensional spatial scattering cluster is satisfied [8–10]. Based on the modeling of visible area of scattering cluster, the coding and decoding structure block diagram of health privacy data coding inside and outside the university physical education class is obtained by using logistics mapping coding and piecewise linear chaotic mapping method, as shown in Figure 3.

### 2.2. Analysis of Data Structure Characteristics

Arithmetic coding is used as it is one of the main algorithms of image compression. It is not only a lossless data compression method, but also an entropy coding method. Other entropy coding methods usually divide the input message into symbols and then encode each symbol, while arithmetic coding directly encodes the entire input message into a number, a decimal *n* satisfying (0.0 ≤ *n* < 1.0), and uses quantitative feature analysis. According to the China Securities Association, quantitative trading refers to a trading method that uses a rigorous and complex mathematical or statistical model, with the help of computer, and through the analysis of a large number of historical data, selects an investment method with excess return on probability, and executes it directly by computer. Quantitative trading has a strong objectivity at the transaction execution level, but in essence, its strategic thinking, investment logic, market selection, and even when to start and stop the operation of the computer are all preselected by investors, which make it a highly subjective trading method. The blockchain scheduling and adaptive control of health privacy data inside and outside the university physical education class are carried out [11]. Combined with public key coding configuration and vector quantization coding, the scattering cluster sequence of health privacy data inside and outside the university physical education class is obtained as Χ=*x*_1_, *x*_2_,…, *x*_*n*_. Turbo code is used to encode and modulate, and the retransmission key of health privacy data inside and outside the university physical education class is expressed as •**RkeyGen**(param, rsk_ID_*i*__, ID_*i*_, ID_*j*_). Combined with nonlinear balanced scheduling, the block feature matching set *S*_*n*_=*x*_1_+*x*_2_+⋯+*x*_*n*_ is obtained [12]. The logarithmic function of this encryption interval of health privacy data inside and outside the university physical education class is as follows:

(1) $$\begin{array}{c} I^{i}=f^{-1}\left(x\right)\left(I^{i+1}\right)\\ \text{size}\left(I^{i}\right)=P_{i}\text{size}\left(I^{i+1}\right), \end{array}$$

where *I*^*i*+1^ is the mutual information and *f*(*x*) is the state objective function of scattering cluster N after the mth scattering. Assuming that the N-dimensional message vector generated by the source S is represented by *x*=(*x*_1_, *x*_2_,…, *x*_*n*_), based on the fitness function *x*_*i*_=2*ε*_*i*_ − 1 analysis of Q cycles, the spatial dynamic matching function of health privacy data coding inside and outside the university physical education class is $S_{\text{obs}}=\left|S_{n}\right|/\sqrt{n}$ by using S transformation, and the linear frequency modulation function for outputting health privacy data inside and outside the university physical education class is obtained by using random coding modulation:

(2) $$\begin{array}{c} \text{size}\left(I^{1}\right)=\Pi_{i=1}^{M}P\left(s_{i}\in S\right)\\ =\Pi_{n=1}^{N}{\left(P_{n}\right)}^{\text{card}\left\{s_{i}|s_{i}=S_{n}\right\}}\\ =\Pi_{n=1}^{N}{\left(P_{n}\right)}^{P_{n}M}, \end{array}$$

where *S* is the broadband true delay energy signal, *s*_*i*_ is the homomorphic key, *P*_*n*_ is the geometric information entropy, and *M* is the encrypted unstructured characteristic value and it is encrypted as bit sequence. Using the data encryption retransmission mechanism shown in Figure 4, the structural reorganization model of health privacy data inside and outside the university physical education class is established [13].

The article "Blockchain-Based Encryption Method for Internal and External Health Privacy Data of University Physical Education Class" was published in 2022. Journal: J Environ Public Health.

According to the combined control model of encryption and retransmission structure of health privacy data inside and outside the university physical education class shown in Figure 2, linear grouping is carried out according to the coded data [*n*, *k*] [14–16]. In PSK source coding, the coded generator *v*(*x*)=*v*_0_+*v*_1_*x*+*v*_2_*x*^2^ ⋯ +*v*_*n*−*k*_*x*^*n*−*k*^ of mixed encryption of the blockchain of health privacy data inside and outside the university physical education class is obtained. Under the combined coded re-signing mode, the following results are obtained:

(3) $$\begin{array}{c} -{\text{log}}_{2}\left(\text{size}\left(I^{1}\right)\right)=-\sum_{n=1}^{N}P_{n}M{\text{log}}_{2}\left(P_{n}\right)=M\cdot H, \end{array}$$

where *I* is the data encryption bit rate, *P*_*n*_ is the public key protocol authorized by the key, *M* is the private parameter, and *H* is the dynamic characteristic value of the public key. According to the above analysis of the structural characteristics of the health privacy data inside and outside the university physical education class, the encryption key in the process of health privacy data transmission inside and outside the university physical education class is designed by detecting the frequency of compressed coding symbols, combining the public key coding configuration and vector quantization coding method [17]. The discrete key transmission sequence of health privacy data inside and outside the university physical education class is constructed by using the natural mode expansion sequence of chaotic logistics, and the feature decomposition model of health privacy data storage inside and outside the university physical education class is established by using the method of random linear feature detection, as shown in Figure 5.

## 3. Optimizing the Storage and Scheduling of Health Privacy Data inside and outside the University Physical Education Class

### 3.1. Blockchain Hybrid Encryption Algorithm

In view of the security threat of quantum computing to blockchain ciphers and the long-term security challenge to blockchain systems, the design theory of blockchain cipher algorithms with anti-quantum computing capability is studied, and blockchain cipher algorithms such as data encryption and digital signature that can resist quantum attacks are designed. Blockchain cryptographic protocols such as identity authentication, secure communication, and secure consensus that can resist quantum attacks are designed. The anti-quantum security blockchain system design theory and data security storage technology are researched and the anti-quantum security blockchain prototype system design method proposed, followed by researching on the fast and secure implementation technology of anti-quantum security public key cryptosystem and studying the solution for migration from the existing cryptographic technology to the anti-quantum computing cryptographic technology in the blockchain.

The article "Blockchain-Based Encryption Method for Internal and External Health Privacy Data of University Physical Education Class" was published in 2022. Journal: J Environ Public Health.

The blockchain hybrid encryption algorithm is used to design the encryption key of health privacy data inside and outside the university physical education class. In the process of cyclic code displacement [18], the bilinear mapping of data encryption is given as: *x*_*i*,*b*_ =  *χ*_*i*,*b*_ − *δ*_*i*,*b*_(1 ≤ *i* ≤ *β*). The private key of blockchain hybrid encryption is: *δ*_*i*,*b*_ =  [*χ*_*i*,*b*_]_*π*_+*ξ*_*i*,*b*_ · *π* − *CRT*_*p*_*m*,*n*__(2*r*_*i*,*b*,*m*,*n*_)_1≤*m*,*n*≤*μ*_, *r*_*i*,*b*,*m*,*n*_ ← *ℤ*∩(−2^*φ*′−1^, 2^*φ*′−1^)， *ξ*_*i*,*b*_ ← *ℤ*∩[0, 2^*λ*+  log_2_(*μ*^2^)+*μ*^2^·*η*^/*π*).

In the complete set of attributes of blockchain hybrid encryption key, a retransmission scheme is given. The generation algorithm of user key is described as *x*′_*i*,*b*_ =  *χ*_*i*,*b*_′ − *δ*_*i*,*b*_′(1 ≤ *i* ≤ *μ*), and the throughput rate of encryption scheme is *δ*′_*i*,*b*_ =  [*χ*′_*i*,*b*_]_*π*_+*ξ*′_*i*,*b*_ · *π* − *CRT*_*p*_*m*,*n*__(2*r*′_*i*,*b*,*m*,*n*_)_1≤*m*,*n*≤*μ*_, *r*′_*i*,*b*,*m*,*n*_ ← *ℤ*∩(−2^*φ*^, 2^*φ*^). The encrypted data is shared to the private key through the public channel, and the identification bit is: *ξ*′_*i*,*b*_ ← *ℤ*∩[0, 2^*λ*+  log_2_(*μ*^2^)+*μ*^2^·*η*^/*π*).

Based on the error correction redundancy logout method, the security parameters of the input key are given as follows: Π_*i*,*b*_ =  *χ*_*i*,*b*_^Π^ − *δ*_*i*,*b*_^Π^(1 ≤ *i* ≤ *μ*), where *δ*_*i*,*b*_^Π^ =  [*χ*_*i*,*b*_^Π^]_*π*_+*ξ*_*i*,*b*_^Π^ · *π* − *CRT*_*p*_*m*,*n*__(2*ϖ*_*i*,*b*,*m*,*n*_+*δ*_*i*,*b*,*m*,*n*_ · 2^*φ*′+1^)_1≤*m*,*n*≤*μ*_; the output ciphertext protocol is: *ϖ*_*i*,*b*,*m*,*n*_ ← *ℤ*∩(−2^*φ*^, 2^*φ*^), *ξ*_*i*,*b*,*m*,*n*_^Π^ ← *ℤ*∩[0, 2^*λ*+2  log_2_(*μ*)+*μ*^2^·*η*^/*π*).

The user is made to convert the public key of the key: *pk*^*∗*^=〈*x*_0_, *se*_1_, (*δ*_*i*,*b*_)_1≤*i*≤*β*,0≤*b*≤1_, (*δ*_*i*,*b*_′)_1≤*i*≤*μ*,0≤*b*≤1_, (*δ*_*i*,*b*_^Π^)_1≤*i*≤*μ*,0≤*b*≤1_〉, according to the corresponding private parameter *x*_*i*,*b*_, *x*′_*i*,*b*_, Π_*i*,*b*_, by optimizing the construction of sparse set; the private key protocol of edge data is: *sk*^*∗*^=(*p*_*i*,*j*_)_1≤*i*,*j*≤*μ*_.

To encrypt (*pk*, *m*_*i*,*j*_ ∈ {0,1}^*μ*×*μ*^), the security parameter characteristics of Turbo code are analyzed, and the encryption key obtained is: *b*=(*b*_*i*,*j*_)_0≤*i*,*j*≤*β*_ ∈ (−2^*α*^, 2^*α*^)^*β*×*β*^ and *b*=(*b*′_*i*,*j*_)_1≤*i*,*j*≤*μ*_ ∈ (−2^*α*′^, 2^*α*′^)^*μ*×*μ*^; the source coding feature quantity is recovered to obtain the output ciphertext: $c^{*}={\left[\sum_{1\leq i,j\leq \mu }m_{i,j}\cdot x_{i,0}^{\prime }\cdot x_{j,1}^{\prime }+\sum_{1\leq i,j\leq \mu }b_{i,j}^{\prime }\cdot \Pi_{i,0}\cdot \Pi_{j,1}+\sum_{1\leq i,j\leq \beta }b_{i,j}\cdot x_{i,0}\cdot x_{j,1}\right]}_{x_{0}}$.

The article "Blockchain-Based Encryption Method for Internal and External Health Privacy Data of University Physical Education Class" was published in 2022. Journal: J Environ Public Health.

To decrypt (*sk*, *c*^*∗*^, *z*), cyclic code displacement parameters are output to obtain information source parameters: $\overset{⟶}{m}=\left(m_{i\text{,}j}\right)$, where *m*_*i*,*j*_ ← [*c*^*∗*^]_*p*_*i*,*j*__, 1 ≤ *i*, *j* ≤ *μ*.

With encrypted retransmission, bit rate of data points is: *x*_*i*_′ mod *p*_*j*_=2*r*_*i*,*j*_′+*δ*_*i*,*j*_; add (*pk*, *c*_1_^*∗*^, *c*_2_^*∗*^). Bus transmission data parameters are: *c*_1_^*∗*^+*c*_2_^*∗*^ mod *x*_0_.

With encryption algorithm, (*pk*, *m*_*i*,*j*_ ∈ {0,1}^*μ*×*μ*^)_1≤*i*,*j*≤*μ*_ is encrypted. The generated ciphertext is *c*, the symbol frequency detection output characteristic quantity is: *c*_1_^*∗*^ · *c*_2_^*∗*^ mod *x*_0_, and the encrypted data becomes: *c* mod *p*_*i*,*j*_=*C*^†^(*c*_1_ mod *p*_*i*,*j*_,…, *c*_*t*_ mod *p*_*i*,*j*_). Introducing blockchain hybrid encryption technology, the coding structure of stop and wait encrypted output is shown in Figure 6.

According to the above analysis, the blockchain hybrid encryption algorithm is used to design the encryption key of the health privacy data inside and outside the university physical education class, and the arithmetic code is embedded in the encryption system to design the multichannel secure transmission [19–22].

### 3.2. Multichannel Secure Transmission of Data

A method for transmitting data such as audio/video (AV) data over multiple channels includes selecting data and encrypting information, and encrypting the data with the encrypted information to generate encrypted data. The encrypted information is divided into several parts. The encrypted data is transmitted using at least one of the plurality of channels, and at least some portions of the encrypted information are transmitted on at least one channel other than the channel on which the encrypted data is transmitted More generally, the encrypted data is transmitted on one channel, and the encrypted information is divided and transmitted on several other channels.

The encryption sparse expression method is introduced to establish a dynamic detection factor analysis model of health privacy data transmission inside and outside the university physical education class. The inverse function of *f* (*x*) is used to store the scheduling value, and coupling vectors of health privacy data inside and outside the university physical education class *b*=(*b*_*i*,*j*_)_0≤*i*,*j*≤*β*_ ∈ (−2^*α*^, 2^*α*^)^*β*×*β*^ and *b*=(*b*_*i*,*j*_′)_1≤*i*,*j*≤*μ*_ ∈ (−2^*α*′^, 2^*α*′^)^*μ*×*μ*^ satisfy

(4) $$\begin{array}{c} c=b\times \sum_{1\leq i,j\leq \beta }b_{i,j}\cdot x_{i,0}\cdot x_{j,1}. \end{array}$$

According to the chaotic coding scheme of logistics [23], a multichannel output model of network data is established. The multichannel transmission feature sequence is: *s*={*s*_*i*_, *i*=1 … *M|s*_*i*_ ∈ *S*}; key parameters are

(5) $$\begin{array}{c} P_{n}=\frac{1}{M}\text{card}\left\{s_{i}|s_{i}=S_{n}\right\}. \end{array}$$

Among them, *S*_*n*_ represents the transmission ratio between channels, *M* represents the key sequence block, and a complete ciphertext sequence is obtained. Thus, multichannel secure transmission is achieved through blockchain hybrid encryption [24].

The article "Blockchain-Based Encryption Method for Internal and External Health Privacy Data of University Physical Education Class" was published in 2022. Journal: J Environ Public Health.

Based on key inquiry, the output key forgery feature quantity is SD. Based on the above analysis, the bit sequence output by blockchain hybrid encryption is circularly shifted to realize the storage and scheduling of health and privacy data inside and outside the university physical education class. The implementation process is shown in Figure 7 [25].

As shown in Figure 7, the storage and scheduling process of health privacy data inside and outside college physical education classes mainly starts with formulating a homomorphic public key encryption mechanism, designing an encryption key, and then designing a decryption key according to the length of the output data packet. On this basis, the characteristic distribution of encrypted bit sequence is determined, the symbol frequency is detected according to the distribution results, the key is filled, and the optimization of data encryption is realized, so as to complete the storage and scheduling of health privacy data inside and outside college physical education classes and also the research on the encryption method of health privacy data inside and outside college physical education classes based on blockchain.

## 4. Simulation Experiment

In order to test the performance of this method in realizing the storage and scheduling of health and privacy data inside and outside the university physical education class, a simulation experiment was conducted. The calculation theory for the full life cycle protection of privacy information selects the health privacy data inside and outside college physical education classes as the test object, uses MATLAB simulation to get the information before and after storage scheduling, compares it, and determines the effectiveness of the method against statistical attacks through information distribution. Under normal circumstances, if the information is evenly distributed and flat, it is judged that the proposed method has good antistatistical characteristics; and if on the contrary, the proposed method has poor antistatistical characteristics. The network data sample length is 1200, the data transmission time interval is 0.37 s, the bandwidth is 45 kHz, and the parameters of multichannel transmission are shown in Table 1.

The article "Blockchain-Based Encryption Method for Internal and External Health Privacy Data of University Physical Education Class" was published in 2022. Journal: J Environ Public Health.

The number of layers of health privacy inside and outside the university of physical education class is set as follows: the confidence of data encryption is 0.869, and the circular displacement of health privacy data inside and outside the university of physical education class is 5.48. See Table 2 for the feature distribution of encrypted data.

According to the parameter settings in Tables 1 and 2, the encrypted storage design of health privacy data inside and outside the university physical education class is carried out [26]. The channel dynamic characteristic parameters are selected to obtain health privacy data inside and outside the university physical education class, as shown in Figure 8.

It can be seen from Figure 8 that for three different encrypted data samples, the time domain waveform distribution of health privacy data inside and outside college physical education classes is relatively uniform, with good results. Taking the time domain waveform data of health privacy data inside and outside college physical education classes in Figure 8 as the test object, under the test environment, through MATLAB simulation, the data security encrypted transmission output of the proposed method is calculated and the encrypted output results obtained, as shown in Figure 9.

By analyzing Figure 9, we can see that the recessive ability of using this method to encrypt health privacy data inside and outside college physical education classes is good, the level of scrambling is high, and the three different encrypted data samples show a good state. The antiattack ability of this method, reference [4] method, and reference [5] method is tested. The encryption performance is shown in Table 3.

According to the comparison results in Table 3, compared with the methods in reference [4] and reference [5], the recognition degree of this method is as high as 97.62%, and the time cost is only 0.43 s. Its antiattack ability is good, the encryption performance is good, and the recognition ability and secure transmission ability of data are improved. The reason is that in the process of multichannel secure transmission of data, the method in this article uses at least one of the multiple channels to transmit the encrypted data and transmits the encrypted data on one channel, and the encrypted information is divided and transmitted on several other channels, which is conducive to enhancing the performance of the method in this article.

To sum up, the encryption method of health privacy data inside and outside college physical education classes based on blockchain has good recessive ability, high scrambling level, strong antiattack ability, and good encryption performance.

The article "Blockchain-Based Encryption Method for Internal and External Health Privacy Data of University Physical Education Class" was published in 2022. Journal: J Environ Public Health.

## 5. Conclusions

Through coding modulation and key control methods, the storage and scheduling of health privacy data inside and outside college physical education classes are realized. This article proposes a storage and scheduling method of health privacy data inside and outside college physical education classes based on blockchain hybrid encryption. The following conclusions are obtained through the study:

1. The time domain waveform distribution of health privacy data inside and outside college physical education classes is relatively uniform
2. This method has better implicit ability and higher scrambling level in storing and scheduling health privacy data inside and outside college physical education classes
3. This method has good security and strong antiattack ability in storing and scheduling health privacy data inside and outside college physical education classes

## Figures and Tables

**Figure 1:** Array direction flowchart.

**Figure 2:** Broadband delay construction flow chart.

**Figure 3:** Block diagram of coding and decoding structure of health privacy data coding inside and outside the university physical education class. (a) Coding process of health privacy data inside and outside universities in physical education class. (b) Decoding process of health privacy data inside and outside the university physical education class.

**Figure 4:** Encryption and retransmission structure of health privacy data inside and outside the university physical education class.

**Figure 5:** Feature decomposition model of health privacy data storage inside and outside the university physical education class.

**Figure 6:** Coding structure of health privacy data inside and outside the university physical education class.

**Figure 7:** Implementation process of encryption of health privacy data inside and outside the university physical education class.

**Figure 8:** Time domain waveform of health privacy data inside and outside the university physical education class. (a) Encrypted data sample 1. (b) Encrypted data sample 2. (c) Encrypted data sample 3.

**Figure 9:** Data encryption output. (a) Encrypted data sample 1. (b) Encrypted data sample 2. (c) Encrypted data sample 3.

**Table 1:** Parameter setting.

Parameter	SNR (dB)	Key threshold	Confidence level
Channel 1	18.813	0.333	0.472
Channel 2	71.533	0.330	0.418
Channel 3	65.007	0.338	0.454
Channel 4	69.143	0.347	0.465
Channel 5	29.342	0.349	0.436
Channel 6	26.128	0.394	0.402
Channel 7	46.403	0.363	0.416
Channel 8	4.966	0.383	0.421

**Table 2:** Characteristic distribution of encrypted data.

Parameter	Matching degree	Similarity	Length (Gbit)
Dataset1	2.7450	4.610	12.179
Dataset2	2.3951	4.466	12.112
Dataset3	2.4773	4.731	12.423
Dataset4	8.1654	4.019	12.333
Dataset5	4.1530	4.334	12.420
Dataset6	7.3042	4.193	12.332
Dataset7	9.1713	4.990	12.468
Dataset8	6.2919	4.262	12.969

The article "Blockchain-Based Encryption Method for Internal and External Health Privacy Data of University Physical Education Class" was published in 2022. Journal: J Environ Public Health.

**Table 3:** Comparison of encryption performance.

Method	Leakage probability	Deciphering bit length (Kbit)	Recognition degree (%)	Time expenditure (s)
Methods of this article	0.056	1.21	97.62	0.43
Reference [4]	0.085	9.56	86.34	0.65
Reference [5]	0.093	12.48	91.55	1.79

## Data Availability

The raw data supporting the conclusions of this article will be made available by the authors, without undue reservation.
